# Efficacy of Super-Mini-PCNL and Ureteroscopy in Kidney Stone Sufferers and Risk Factors of Postoperative Infection

This article has been retracted.

**DOI:** 10.1155/2022/4733329

**Published:** 2022-03-08

**Authors:** Wenbing Yuan, Yingyi Li, Yu Dai, Cheng Luo, Hui Zhang, Haijun Xiong

**Affiliations:** Urology Surgery, Baoji City People's Hospital, Baoji 721000, Shannxi Province, China

## Abstract

To investigate the efficacy of super-mini-PCNL (SMP) and ureteroscopy in kidney stone (KS) sufferers and learn the risk factors of postoperative infection. A retrospective analysis was performed on 180 KS sufferers who were diagnosed and treated in our hospital from May 2019 to May 2021. They were enrolled into an observation group (OG, *n* = 104) and a control group (CG, *n* = 76) based on different treatment methods. Therein, the former was treated with SMP, while the latter was treated with ureteroscopy. The operation time, blood loss, hospital stay, recent stone-free rate (one week after operation), changes of serum creatinine (SCr), blood urea nitrogen (BUN), and cystatin C (CysC) levels before and after operation and complications were compared. Those sufferers were assigned to infected and uninfected groups based on their postoperative infection. The risk factors were assessed through logistic regression, and the model formula was established. The predictive value of this model for infection was tested through RO. Compared with CG, the operation time of the OG was longer, the blood loss and hospital stay were lower (*P* < 0.05), and the stone-free rate was higher (*P* < 0.05). Renal function indexes before and after treatment (*P* > 0.05) and postoperative complications revealed no significant difference (*P* > 0.05). Logistic regression analysis manifested that preoperative urinary tract infection (OR: 4.690, 95% CI: 1.170–18.802), preoperative blood glucose level (OR: 11.188, 95% CI: 2.106–59.442), positive urine culture (OR: 10.931, 95% CI: 2.453–48.705), and infectious stones (OR: 3.951, 95% CI: 1.020–15.300) were independently related to infection. The risk prediction equation is logit(*p*)=−8.913+1.545 × *X*1+2.415 × *X*2+2.392 × *X*3+1.374 × *X*4, with a goodness-of-fit value of 0.545. The AUC is 0.930, so SMP is superior to ureteroscopy in KS sufferers. Preoperative urinary tract infection, preoperative blood glucose level, positive urine culture, and infectious stones are independently related to infection.

## 1. Introduction

### 1.1. Incidence of Renal Calculi

Kidney stone (KS) is one of the familiar diseases of urinary system. Statistics show that 5–15% of the global population is plagued by KS [1]. A survey found that the number of KS sufferers increased by 70% from 1994 to 2010 [2]. In another study, from 1992 to 2009, the rate of visits to emergency departments for stones increased by 91% [3]. Not only that, due to the mounting sufferers from population, obesity and metabolic syndrome (independent risk factors for KS), the annual cost of treatment in the US exceeds $10 billion in the medicare system [4]. Although most stones will not have long-term consequences, it was once thought that KS is related to chronic kidney disease (CKD) [5]. In addition, the recurrence rate is very high: 50% within 5–10 years and 75% within 20 years [6]. Thus, choosing an effective treatment plan is the key to improve the current situation.

### 1.2. Progress in the Treatment of Renal Calculi

Chinese urology guidelines for diagnosis and treatment believe that conservative treatment can be considered for stone diameter＜0.4 cm, and 90% of them may pass spontaneously; however, for stones <0.6 cm, with a smooth surface, no obstruction of the lower urinary tract, and staying in the local area for less than 2 weeks, drug stone removal is the first choice [7], but it takes a long time so that most patients cannot bear the pain caused by the disease. Clinically, there are many surgical treatment schemes for KS. There are mainly five schemes: traditional open lithotripsy, extracorporeal shock wave lithotripsy (ESWL), laparoscopic lithotripsy, percutaneous nephrolithotomy (PCNL), and flexible ureteroscopic lithotripsy (FURL), among which ESWL and PCNL are still in the front line [8]. PCNL still plays a vital role in urology surgery, which protects a large number of KS sufferers against open surgery [9]. Although PCNL has a high stone-free rate, patients need massive transfusions during operations, and the duration is long, which will inevitably increase the occurrence of complications such as vital organ injury and hemopneumothorax [10]. As efficacy develops, super-mini-PCNL (SMP) has been generalized in clinical practice [11]. The SMP channel is usually F10-14. Comparatively speaking, such a small channel is less traumatic and bleeding. Nowadays, new ureteroscopes and related auxiliary equipment are also developing continuously, which not only improves safety and shortens the operation time, but also reduces the incidence of complications, particularly bleeding. Ureteroscopy also achieved a higher stone-free rate than SMP [12], which has become an alternative surgical scheme for clinicians.

*Purpose of the Study.* But for surgical treatment of stones ≤2 cm, SMP or ureteroscopy is still disputed. In this research, we retrospectively analyzed the influence of SMP and ureteroscopy on the efficacy of KS sufferers and assessed the risk factors of postoperative infection by logistic regression, so as to provide a reference for clinical surgical treatment.

## 2. Methods and Data

### 2.1. Clinical Data of Patients

A retrospective analysis was performed on 180 KS sufferers diagnosed and treated in our hospital from May 2019 to May 2021. In the light of different treatment methods, they were assigned to an observation group (OG, *n* = 104) and a control group (CG, *n* = 76). Therein, the former was treated with SMP, while the latter was treated with ureteroscopy with the consent of the Medical Ethics Committee.

### 2.2. Inclusion and Exclusion Criteria

#### 2.2.1. Inclusion Criteria

The inclusion criteria were as follows: KS sufferers with imaging analysis, intravenous pyelography, and abdominal plain film (diameter ≤2 cm); it was ineffective after ESWL; and patients or their families who signed an informed consent form.

#### 2.2.2. Exclusion Criteria

The exclusion criteria were as follows: those who were intolerable about this operation or drugs; those complicated with tumor or congenital organ defects; the ureter has anatomical malformations such as stenosis and ectopia; pregnant women; and those aged <18 years old.

### 2.3. Surgical Treatment Plan

The treatment plan of SMP is as follows: anesthetized sufferers were in the lithotomy position; the affected side was inserted into a retrograde ureteroscope to guide them to a prone position under the cystoscope. Under B-ultrasound, the renal calyces were punctured with F13 SMP kits, the delaser optical fiber was placed, and an incision was made in the skin to expand it to F14 along the guide wire. The metal sheath was retained, a percutaneous nephrolithotomy channel was created, and then a ureteroscope or human standard nephrolithotomy was put in. An ultrasonic lithotripsy system was used for lithotripsy (frequency 25 Hz/energy 1.0 J/power 20 W) to obtain stones < 3 mm. With normal saline, the crushed stones were washed out through the sheath along the inner wall of the sheath, and the F6 double-J tube was maintained; 1–4 weeks later, the nephrostomy tube was removed.

The treatment plan of ureteroscope is as follows: sufferers were in the same position. The ureter superfine nephroscope was put in, the F5 tube was set up in the renal pelvis to dilate the ureter, 0.035 < 3 mm ultrasmooth guide wire was employed to retain and send it to the ureteroscope, and a 200 *μ*m smooth guide wire was placed into the soft endoscope sheath to locate stones (frequency 15–20 Hz/energy 1.0–1.5 J/power 10–25 W). The stones were crushed until the diameter <3 mm. The F5 double-J tube was maintained after the stone fragments were collected by the stone extraction basket and pulled out 1–4 weeks later, and the F14 tube was removed after nephrostomy. Antibiotics were routinely utilized in both groups after operations to prevent infection.

### 2.4. Clinical Index Test

Peripheral blood (5 mL) was collected, then isolated at 3000 rpm/min, and centrifuged for 10 min to obtain the supernatant. Serum creatinine (SCr), blood urea nitrogen (BUN), and cystatin C (CysC) levels were tested. CysC was tested by enhanced immunoturbidimetry, BUN by ELISA, and SCr by the picric acid method, under the Beckman 5800 automatic biochemical analyzer. All the CysC, BUN, and SCr kits were offered by the manufacturers, and all the steps were based on the instructions and were completed by the same inspection team in line with the aseptic operation rules.

### 2.5. Outcome Measures

The primary outcome measures were as follows: the perioperative indicator changes (operation time, blood loss, and hospital stay) and stone-free rate one week after operation (clearance rate = stone-free rate/primary stone quantity × 100%) of both groups were compared. The renal function, such as SCr, BUN, and CysC, was compared before and after the operation.

The secondary outcome measures were as follows: the clinical data (gender, age, stone diameter, past medical history (hypertension and diabetes), smoking, and alcoholism), complications (infection, delayed bleeding, fever, and urinary fistula), and the overall incidence were tested (total incidence = cases/total number × 100%). Sufferers were assigned to the infected (*n* = 15) or uninfected groups (*n* = 166) based on their infection. The risk factors were assessed through logistic regression.

### 2.6. Statistical Analysis

Data were processed via SPSS 20.0 and then visualized by GraphPad Prism 8 software. Specifically, the independent sample *t*-test was conducted for intergroup comparison and the paired *t*-test for intragroup comparison, both expressed in *t*. The rank-sum test was utilized for ranked data expressed by *Z*, and the chi-square test was performed on counting data. The risk factors were assessed via logistic regression (forward was utilized for univariate analysis and backward LR for multivariate analysis). The Hosmer–Lemeshow test was used to correct the discrimination and goodness-of-fit of the ROC curve model. *P* < 0.05 was statistically different.

## 3. Results

### 3.1. Clinical Data Comparison

It was found that there was no statistical difference in gender, age, stone diameter, previous medical history, smoking, and alcoholism history between both groups (Table 1; *P* > 0.05).

### 3.2. Comparison of Perioperative Indicators

It was found that both the operation time and hospitalization time of patients in the CG were higher than those in the OG, with statistical differences (Figures 1(a) and 1(b); *P* < 0.001). Besides, the blood loss in the CG was higher (Figure 1(c); *P* < 0.001).

### 3.3. Comparison of Recent Stone-Free Rates

The recent stone-free rate of the OG was higher than that of the CG, with statistical differences (Table 2; *P* < 0.05).

### 3.4. Renal Function Changes

It was found that the BUN, SCr, and CysC levels in both groups were lower after treatment than before treatment, with statistical differences (*P* < 0.001). But the three levels revealed no marked difference after the operation (Figures 2(a)–2(c); *P* > 0.05).

### 3.5. Comparison of Postoperative Complications

CG had 6 cases of postoperative infection, 3 of delayed bleeding, 2 of fever, and 2 of urinary fistula. While in the OG, there were 9 cases of postoperative infection, 3 of delayed bleeding, 1 of fever, and 1 of urinary fistula. There was no difference in the incidence of complications between the two groups (*P* > 0.05). And the total incidence rate of both groups also showed no statistical difference (Table 3; *P* > 0.05).

### 3.6. Analysis of Infection Risk Factors

Finally, sufferers were assigned to the infected (*n* = 15) and uninfected groups (*n* = 166) based on their infection, and clinical data were collected (Table 4). Signal and multivariant logistic regression demonstrated that urinary tract infection (OR: 4.690, 95% CI: 1.170–18.802), preoperative blood glucose level (OR: 11.188, 95% CI: 2.106–59.442), positive urine culture (OR: 10.931, 95% CI: 2.453–48.705), and infectious stones (OR: 3.951, 95% CI: 1.020–15.300) were independent risk factors for infection (Tables 5 and 6; *P* < 0.05). The risk prediction equation was established based on multivariate logistic regression: logit(*p*)=−8.913+1.545 × *X*1+2.415 × *X*2+2.392 × *X*3+1.374 × *X*4, and the regression equation goodness-of-fit was tested through the Hosmer–Lemeshow test (*P*=0.545). The established model was used to test the AUC of postoperative infection in KS sufferers with a value of 0.930 (specificity: 93.33% and sensitivity: 81.81%) (Figure 3 and Table 7). According to the risk prediction score model established, the probability of postoperative infection in patients with infectious stones is 60.00%, and that of ineffectiveness after treatment in RA patients whose disease course is less than 2 years is 80.60%.

## 4. Discussion

As living standards changes and dietary structure develops, KS incidence has been growing. It is a human mineralized disease with a complicated etiology [13]. Data statistics reveal that KS is highly likely to relapse, and the 5–10-year recurrence rate has reached more than 50% [14]. Its formation cause is vague, which is affected not only by individual factors such as urinary tract, metabolism, and gene abnormalities, but also by the environment ( such as geography, climate, and diet) [15]. Medication is a frequently used treatment at present [16]. But due to the slow onset and long treatment period, it is difficult to achieve the desired effect, which makes the surgical treatment of stones popular [17]. Clinically, the traditional treatment scheme for stones is mainly open surgery. However, open surgery has caused great trauma to patients, sometimes requiring multiple operations to remove stones, and the probability of postoperative complications is high, causing serious damage to renal function [18]. Therefore, these two treatment schemes are gradually being replaced by minimally invasive surgery.

ESWL is noninvasive and repeatable, with no anesthesia, low cost, and no wound on the body surface. It is also an outpatient treatment. It can crush stones in any part of the kidney [19]. Admittedly, it is not completely harmless. It can cause irreversible complete loss of renal function, and infection, bleeding, irreversible damage of renal function, and renal parenchyma may occur during treatment [20]. Moreover, the efficacy is relevant to many factors such as the shape and size of stones, with a high recurrence rate.

SMP and ureteroscopy have become the main surgical schemes for clinical treatment. Nevertheless, there is still controversy about the two schemes. To this end, we compared the effects of the two on the efficacy of patients. BUN is a proteinmetabolism product, which will obviously increase when the glomerular filtration rate is reduced to 50% of normal [21]. SCr is a crucial indicator of renal excretion function. When renal function is damaged, its content in human body will dramatically increase. The sensitivity of CysC is extremely high, and its content will rise rapidly in the early stage of kidney injury. The abovementioned changes of the three are essential criteria for clinical evaluation of renal function. Furthermore, we discovered the renal function indexes decreased after treatment with no difference. Moreover, there is no difference in the incidence of postoperative complications, which suggests that the two surgical schemes can substantially improve the prognosis of patients with renal injury without increasing the incidence of postoperative complications. The operation time and hospital stay of SMP were shorter than those of ureteroscopy, and the blood loss during the operation was lower. Not only that, the recent stone-free rate of patients treated by SMP was higher. This is largely due to the negative pressure suction system of SMP, which ensures its stone removal efficiency well. With the help of the negative pressure suction device, the crushed stones can be quickly sucked out from the suction sheath to the collection bottle, which improves the removal rate, reduces the use of the net basket and the lithotripsy forceps, and accelerates the operation speed. In the process of ureteroscopy, only a 200 *μ*m holmium laser is adopted for lithotripsy; the instrument is single, and the efficiency is low, which is greatly influenced by the stone hardness.

Postoperative infection is the challenge for all surgical patients after an operation. This research examined the postoperative infection of patients. Logistic regression analysis manifested that preoperative urinary tract infection, preoperative blood glucose level, positive urine culture, and infectious stones were related to infection. For that, the urinary tract infection process and urinary calculus formation are relevant and complementary, and the presence of urinary tract infection before operation will increase the risk of postoperative infection. Higher blood glucose increases plasma osmolality and reduces immunologic cellular activity, thus lowering the body's resistance to pathogenic bacteria and increasing the incidence of infection. Prior research found that positive urine culture and infectious stones were relevant to postoperative infection, which was associated with our results. Therefore, patients should be examined as early as possible before the operation and treated promptly to reduce the risk of infection. Finally, we constructed the risk model of infection prediction based on regression results. By fitting and drawing the ROC curve, we calculated that the area of the model under the curve of infection prediction was 0.930, which was ideal.

We also determined that the efficacy of SMP was better than that of ureteroscopy and analyzed the postoperative infection factors. Nevertheless, this research still has some limitations. Firstly, it is a retrospective study with a limited sample size, so it is impossible to increase the comparability of the research like the random control group experiment in sample selection. Secondly, patients cannot be followed up for long periods. It is well known that KS is likely to recur, but it is indistinct whether the two kinds of surgery affect postoperative recurrence. Thus, we hope to conduct randomized controlled trials and perfect our findings on inflammation through long-term follow-up.

To sum up, the efficacy of SMP in treating KS sufferers is better than that of ureteroscopy. Preoperative urinary tract infection, preoperative blood glucose level, positive urine culture, and infectious stones are independently related to infection.

## Figures and Tables

**Figure 1:** Perioperative indicator comparison. (a) Comparison of operation time between both groups. (b) Comparison of hospital stay between both groups. (c) Comparison of intraoperative blood loss between both groups. ^*∗∗∗*^*P* < 0.001.

**Figure 2:** Renal function indexes of patients before and after operation. (a) Changes of BUN levels before and after treatment. (b) Changes of SCr levels before and after treatment. (c) Changes of CysC levels before and after treatment. ^*∗∗∗*^*P* < 0.001.

**Figure 3:** ROC curve of predicting combined indicators of postoperative infection in patients.

**Table 1:** Basic figures (*n* (%)).

Factor		CG (*n* = 76)	OG (*n* = 104)	*P* value
Gender				0.348
	Male (*n* = 116)	46 (60.53)	70 (67.31)	
	Female (*n* = 64)	30 (39.47)	34 (32.69)	

Age				0.676
	≥40 years old (*n* = 82)	36 (47.37)	46 (44.23)	
	<40 years old (*n* = 98)	40 (52.63)	58 (55.77)	

Stone diameter				0.574
	≥1 cm (*n* = 141)	58 (76.32)	83 (79.81)	
	<1 cm (*n* = 39)	18 (23.68)	21 (20.19)	

Past medical history				
	Diabetes (*n* = 44)	16 (21.05)	28 (25.93)	0.365
	Hypertension (*n* = 61)	25 (32.89)	36 (34.62)	0.810

History of smoking				0.530
	Yes (*n* = 123)	50 (65.79)	73 (70.19)	
	No (*n* = 57)	26 (34.21)	31 (29.81)	

History of alcoholism				0.364
	Yes (*n* = 34)	12 (15.79)	22 (21.15)	
	No (*n* = 146)	64 (84.21)	82 (78.85)	

**Table 2:** Recent stone-free rate (*n* (%)).

Group	Cleared	Not cleared	*χ*2 value	*P* value
CG (*n* = 76)	57 (75.00)	19 (25.00)	7.690	0.006
OG (*n* = 104)	94 (90.38)	10 (9.62)		

**Table 3:** Complications.

Group	Infection	Delayed bleeding	Fever	Urinary fistula	Total incidence rate
CG (*n* = 76)	6 (7.89)	3 (3.94)	2 (2.63)	2 (2.63)	13 (17.11)
OG (*n* = 104)	9 (8.65)	3 (2.88)	1 (0.96)	1 (0.96)	14 (13.46)
*χ*2 value	0.033	0.154	0.747	0.747	0.457
*P* value	0.856	0.695	0.387	0.387	0.499

**Table 4:** Assignment table.

Factor	Assignment
Gender (*X*)	Male = 1, female = 2
Age (*X*)	≥40 = 1, <40 = 2
Diameter of stones (*X*)	≥1 cm = 1, <1 cm = 2
Operation time (*X*)	Raw data are used as continuous variables
History of diabetes (*X*)	Yes = 1, no = 2
History of hypertension (*X*)	Yes = 1, no = 2
Preoperative urinary tract infection (*X*)	Yes = 1, no = 2
Preoperative blood glucose level (*X*)	≥6.1 mmol/L = 1, <6.1 mmol/L = 2
Positive urine culture (*X*)	Yes = 1, no = 2
Infectious stones (*X*)	Yes = 1, no = 2
Infection (*Y*)	Infected = 1, uninfected = 2

**Table 5:** Logistic univariate analysis.

	*β*	S.E	*χ* ^2^ value	*P* value	OR value	95% CI
Sex	0.107	0.571	0.035	0.851	1.113	0.363–3.411
Age	−0.560	0.570	0.966	0.326	0.571	0.187–1.745
Diameter of stones	−0.301	0.614	0.240	0.625	0.740	0.222–2.467
Operation time	0.004	0.020	0.034	0.855	1.004	0.965–1.044
History of diabetes	0.128	0.611	0.044	0.834	1.136	0.343–3.767
History of hypertension	0.486	0.685	0.502	0.478	1.625	0.424–6.221
Preoperative urinary tract infection	1.386	0.572	5.872	0.015	4.000	1.303–12.275
Preoperative blood glucose level	2.538	0.777	10.664	0.001	12.652	2.758–58.031
Positive urine culture	2.337	0.668	12.221	<0.001	10.348	2.792–38.355
Infectious stones	2.118	0.582	13.239	<0.001	8.312	2.656–26.011
Surgical plans	−0.05	0.55	0.008	0.927	0.951	0.323–2.796

**Table 6:** Logistic multivariate analysis.

	Β	S.E	*χ* ^2^ value	*P* value	OR value	95% CI
Preoperative urinary tract infection	1.545	0.708	4.758	0.029	4.690	1.170–18.802
Preoperative blood glucose level	2.415	0.852	8.031	0.005	11.188	2.106–59.442
Positive urine culture	2.392	0.762	9.842	0.002	10.931	2.453–48.705
Infectious stones	1.374	0.691	3.956	0.047	3.951	1.020–15.300

**Table 7:** ROC curve parameters.

Index	Parameter
AUC	0.930
Std. error	0.028
95% CI	0.874–0.985
*P* value	<0.001
Specificity	93.33%
Sensitivity	81.81%
Youden index	75.15%
Cut-off value	> 0.930

*Note.* AUC: area under curve.

## Data Availability

No data were used to support this study.
